# PTBP1 as a Promising Predictor of Poor Prognosis by Regulating Cell Proliferation, Immunosuppression, and Drug Sensitivity in SARC

This article has been retracted.

**DOI:** 10.1155/2022/5687238

**Published:** 2022-05-23

**Authors:** Haiyi Gong, Aimin Jiang, Runyi Jiang, Yao Wang, Dan Zhang, Zhipeng Wu, Jianru Xiao

**Affiliations:** ^1^Department of Orthopedic Oncology, Shanghai Changzheng Hospital, Naval Medical University (The Second Military Medical University), Shanghai, China; ^2^Department of Urology, Shanghai Changhai Hospital, Naval Medical University (The Second Military Medical University), Shanghai, China

## Abstract

**Background:**

Sarcomas (SARC) have been found as rare and heterogeneous malignancies with poor prognosis. PTBP1, belonging to the hnRNPs family, plays an essential role in some biological functions (e.g., pre-mRNA splicing, cell growth, and nervous system development). However, the role of PTBP1 in SARC remains unclear. In this study, the aim was to investigate the potential role of PTBP1 with a focus on SARC.

**Methods:**

The expression, prognostic value, possible biological pathways of PTBP1, and its relationship with immune infiltration and drug sensitivity were comprehensively analyzed based on multiple databases. PTBP1 was further validated in osteosarcoma as the most prominent bone SARC. The expression of PTBP1 was investigated through IHC. The prognostic value of PTBP1 was verified in TARGET-OS databases. CRISPR/Cas9-mediated PTBP1 knockout HOS human osteosarcoma cell lines were used to assess the effect of PTBP1 on cell proliferation, migration, metastasis and cell cycle by CCK-8, Transwell migration, invasion, and FACS experiment.

**Result:**

PTBP1 was highly expressed and significantly correlated with poor prognosis in several cancers, especially in SARC, which was validated in the clinical cohort and osteosarcoma cell lines. The genetic alteration of PTBP1 was found most frequently in SARC. Besides, PTBP1 played a role in oncogenesis and immunity through cell cycle, TGFB, autophagy, and WNT pathways at a pan-cancer level. Knockout of PTBP1 was observed to negatively affect proliferation, migration, metastasis, and cell cycle of osteosarcoma in vitro. Furthermore, PTBP1 was significantly correlated with tumor immune infiltration, DNA methylation, TMB, and MSI in a wide variety of cancers. Moreover, the potential of the expression level of PTBP1 in predicting drug sensitivity was assessed.

**Conclusions:**

PTBP1 is highly expressed and correlated with prognosis and plays a vital pathogenic role in oncogenesis and immune infiltration of various cancers, especially for SARC, which suggests that it may be a promising prognostic marker and therapeutic target in the future.

## 1. Introduction

Sarcomas (SARC) are rare heterogeneous malignancies with over 50 histologic subtypes. They account for approximately 1% of all malignancies and are generally classified as soft tissue sarcoma (STS) and bone sarcoma (BS) [1–3]. The treatment of SARC is still a huge clinical challenge due to their diversity and aggressive biological behavior. Complete surgical resection combined with adjuvant or neoadjuvant radiotherapy is still the main treatment for localized primary SARC. However, many patients still have recurrence and metastasis, partially because SARC has high malignancy and is prone to metastasis [4]. Despite a combination of surgery, systemic radiotherapy, and chemotherapy used for treating metastatic SARC, the median overall survival (OS) of patients does not exceed 2 years [5]. The advent and rapid progress of immunotherapy has raised new hopes for treating SARC [6–10]. Thus, potential prognostic marker and therapeutic target in SARC should be urgently found.

Polypyrimidine Tract-Binding Protein 1 (PTBP1, hnRNP I), a member of the hnRNPs family, can mediate RNA maturation, translocation, localization, and translation. Its aberrant expression has been detected in numerous diseases. The most extensive role of PTBP1 is a major inhibitory splicing factor involved in regulating alternative splicing (AS) of precursor mRNA (pre-mRNA), leading to exon skipping [11]. PTBP1 has been found to be correlated with tumor metastasis, which leads to a poor prognosis in patients [12]. It mediates tumor development by regulating the cellular metabolism [13] and immune response of T/B lymphocytes as a splicing regulator [14, 15], which has an effect on the immune infiltration of tumor cells. PTBP1 plays a wide range of roles in tumorigenesis, so it may be proven as a novel therapeutic target. However, few studies have systematically analyzed PTBP1 from a pan-cancer perspective, and the comprehensive function of PTBP1 in SARC remains unclear.

In this study, the correlation between the expression of PTBP1 and prognosis, genetic alterations, potential biological pathways, immune infiltration, and drug sensitivity in human cancers was comprehensively analyzed using multiple databases, with a focus on SARC. PTBP1 was found to be upregulated, positively correlated with malignant biological behavior, and significantly correlated with poor prognosis for patients with SARC, which was validated in osteosarcoma. We also found that PTBP1 might be potentially involved in signaling pathways that regulated oncogenesis and tumor immunity, and its expression was correlated with DNA damage repair systems, DNA methylation, TMB, and MSI at a pan-cancer level. Our findings reveal that PTBP1 might be a prognostic and immune infiltration marker in numerous cancers, especially in SARC.

## 2. Materials and Methods

### 2.1. Data Source and Processing

Normalized expression profile data, tumor mutational burden (TMB) data, microsatellite instability (MSI) data and clinical information of The Cancer Genome Atlas (TCGA) datasets, normal tissues datasets, and TARGET OS datasets were acquired from University of California Santa Cruz Xena (UCSC Xena; https://xena.ucsc.edu/) and Genotype-tissue expression (GTEx; https://gtexportal.org/home/). Oncomine (https://www.oncomine.org) was adopted to validate the expression difference of PTBP1 in pan-cancer settings, which was a web-based data mining platform assembling 86,733 samples and 715 gene expression datasets [16]. Human protein atlas (HPA; https://www.proteinatlas.org/) database was adopted to assess the difference in the expression of PTBP1 at the protein level in pan-cancer settings. Cancer Cell Line Encyclopedia (CCLE; https://portals.broadinstitute.org/) database was employed to acquire the expression data of the respective tumor cell line. Patients were excluded if they (1) did not have prognostic information and (2) died in 30 days.

The RNA-seq read counts acquired from public databases were employed for differentially expressed gene (DEG) detection, which were converted to transcripts per kilobase million (TPM). The log2 (TPM+1) calculation was conducted for further analyses.

Tumor name abbreviations and corresponding meanings consisted of ACC (adrenocortical carcinoma), BLCA (bladder urothelial carcinoma), BRCA (breast invasive carcinoma), CESC (cervical squamous cell carcinoma and endocervical adenocarcinoma), CHOL (cholangiocarcinoma), COAD (colon adenocarcinoma), COAD (colon adenocarcinoma), READ (rectum adenocarcinoma esophageal carcinoma), DLBC (lymphoid neoplasm diffuse large B-cell lymphoma), ESCA (esophageal carcinoma), GBM (glioblastoma multiforme), HNSC (head and neck squamous cell carcinoma), KICH (kidney chromophobe), KIRC (kidney renal clear cell carcinoma), KIRP (kidney renal papillary cell carcinoma), LAML (acute myeloid leukemia), LGG (brain lower grade glioma), LIHC (liver hepatocellular carcinoma), LUAD (lung adenocarcinoma), LUSC (lung squamous cell carcinoma), MESO (mesothelioma), OV (ovarian serous cystadenocarcinoma), PAAD (pancreatic adenocarcinoma), PCPG (pheochromocytoma and paraganglioma), PRAD (prostate adenocarcinoma), READ (rectum adenocarcinoma), SARC (sarcoma), SKCM (skin cutaneous melanoma), STAD (stomach adenocarcinoma), STES (stomach and esophageal carcinoma), TGCT (testicular germ cell tumors), THCA (thyroid carcinoma), THYM (thymoma), UCEC (uterine corpus endometrial carcinoma), and UVM (uveal melanoma).

### 2.2. Differential Expression Analysis and Validation of PTBP1

The expression of PTBP1 was analyzed in Oncomine database among pan-cancer with *P* < 0.05 and absolute Foldchange > 1.5 as the threshold. The same threshold was adopted to identify differential expression levels of PTBP1 in the TCGA database. The cBioPortal database (https://www.cbioportal.org) was employed to investigate the copy number alteration and mutation landscape of PTBP1 in pan-cancer. Furthermore, the correlation between PTBP1 and methylation level at the locus was investigated among pan-cancer.

### 2.3. Enrichment Analysis of PTBP1

Pearson's correlation between PTBP1 and other mRNA expression retrieved was studied based on the guilt of correlation of s single gene in the expression profile. After the genes were sorted by the level of correlation index between genes and PTBP1, those genes most correlated with the expression of PTBP1 were selected for enrichment analysis. R package “clusterprofiler” was adopted to perform Gene Ontology (GO) analysis, Reactome analysis, Kyoto Encyclopedia of Genes and Genomes (KEGG) analysis, and Gene Set Enrichment Analysis (GSEA) [17].

### 2.4. Assessment of Clinical Significance of the Expression of PTBP1

Clinical characteristics (e.g., the tumor stage and drug sensitivity) were introduced, and the correlation between the expression of PTBP1 and the above characteristics was investigated. Cell Miner (https://discover.nci.nih.gov/cellminer/home.do) and GDSC (https://www.cancerrxgene.org/) database were acquired for IC50 (half maximal inhibitory concentration) and gene expression of cancer cell lines [18, 19].

### 2.5. Differences in TME and Immunotherapy Response

The correlation between the infiltration degree of immune, stromal cells, and the expression of PTBP1 in pan-cancer was analyzed using R package “ESTIMATE”. R package “ggpubr” and “ggcor” was employed for the coexpression analysis of immune-related gene and the expression of PTBP1. R package “CIBERSORT” was used to quantify the immune cell infiltration scores among pan-cancer, and the correlation of the degree of immune cell and the expression of PTBP1 were obtained [20]. In addition, the correlation between Neo antigen count, TMB, MSI, and expression of T cell exhaustion markers genes (PDCD1, TIGIT, CD274, CTLA4, LAG3, CXCL13, LAYN, and HAVCR2), DNA mismatch repair (MMR) system genes (MLH1, MSH2, MSH6, PMS2, and EPCAM), DNA methyltransferase (DNMT1, DNMT2, DNMT3A, and DNMT3B), ESTIMATE scores, and the expression of PTBP1 was analyzed. The immune infiltration scores were obtained using ssGSEA algorithm, and the correlation and difference between immune cell infiltration and the expression level of PTBP1 in SARC were analyzed. The effect of PTBP1 mutation on immune cell infiltration in SARC was validated using TIMER website (https://timer.cistrome.org/) [21].

### 2.6. Statistical Analysis

Differences in the expression of PTBP1 in the public data sets were compared by one-way ANOVA, and differences in clinical information and immune checkpoint inhibitor response between the two different subgroups were compared by Chi-squared test. Differences in overall survival (OS), progression-free interval (PFI), and disease-specific survival (DSS) between the two subgroups were compared by Kaplan-Meier method and log-rank rest. The common cutoff value was the median of the expression of PTBP1, and the cutoff value of TARGET-OS dataset was determined by function “surv_cutpoint” of package “survminer”. The hazard ratios (HRs) were obtained by univariate Cox regression and multiple Cox regression analysis. All *P* values were two-sided; *P* < 0.05 indicated the difference with statistical significance. Adjusted *P* value was obtained by Benjamini-Hochberg (BH) multiple test correction. All data processing, statistical analysis, and plotting were conducted with R 4.0.4 software.

### 2.7. Validation of Different Expression Levels of PTBP1

Immunohistochemical (IHC) staining was performed to validate the expression of PTBP1 in osteosarcoma tumor and adjacent tissues, including 30 osteosarcoma tumor tissues and 12 adjacent tissues from Shanghai Changzheng hospital. IHC staining intensity of PTBP1 was scored by three experienced pathologists. The staining degree was classified into 0 (negative), 1 (weakly positive), 2 (moderately positive), and 3 (strongly positive). Western blotting was performed to validate the expression of PTBP1 among human osteosarcoma cell lines (HOS/MG63/Saos2/U2OS) and hBMSC cell line. PTBP1 antibody (anti-PTBP1 antibody, [EPR9048(B)], (ab133734), Abcam) originated from Abcam Trading Co., LTD.

### 2.8. PTBP1 Biological Function In Vitro

Human bone marrow stromal (mesenchymal) stem cell line hBMSC and human osteosarcoma cell lines (HOS, MG63, Saos2, and U2OS) originated from American Type Culture Collection (ATCC). Cell lines were cultured following the instructions. Cas9/sgRNA of PTBP1 was synthesized by OBiO Technology (Shanghai) Corp., Ltd. Human osteosarcoma cell line HOS was transduced with Cas9 lentiviral particles of sgRNAs. Cells were selected with Puromycin. The specific procedures followed the operation manual of OBiO Technology (Shanghai) Corp., Ltd. RT-PCR and Western blot assay were performed to confirm the knockout efficiency of Cas9 virus. Specific primer sequences included PTBP1 (forward: AGCGCGTGAAGATCCTGTTC; reverse: CAGGGGTGAGTTGCCGTAG), synthesized by Tsingke Biotechnology Co., Ltd., Beijing, China. Cell proliferation, migration, and invasion between HOS and HOS-PTBP1-knockout cell lines were detected by CCK-8 (Cell Counting Kit-8), Transwell migration, and invasion assay. Cell cycle distribution was analyzed by fluorescence-activated cell sorting (FACS) experiment. All experiments were performed as triplicates and repeated at least three times.

## 3. Results

### 3.1. TPBP1 Gene Expression and Survival Analysis

Oncomine database was used to determine the expression of PTBP1 pattern among pan-cancer which revealed that PTBP1 was overexpressed in tumor tissues compared to normal tissues at a pan-cancer level (Figure 1(a)). More nuanced analyses were conducted in cancer tissues vs. normal tissues (Figure 1(b)), as well as cancer vs. paired adjacent tissues using data acquired from TCGA and GTEx cohort (Figure 1(c)). We observed a higher expression level of PTBP1 in BCLA, BRCA, CHOL, COAD, ESCA, HNSC, KIRC, KIRP, LIHC, LUSC, READ, STAD, and UCEC significantly for both comparisons (*P* < 0.05). Further analyses of the expression level of PTBP1 among different clinical stages of cancers showed that PTBP1 was correlated with advanced clinical stage in ACC, ESCA, and KICH, opposite trend in KIRC, MESO, and SKCM (Supplement Figure 1).

As revealed by the univariate Cox regression analysis results, PTBP1 might be a risk factor for the prognosis of ACC, KICH, LGG, LIHC, LUAD, MESO, PRAD, SARC, and SKCM patients, while being a protective factor in KIRC, READ, and THYM (Figure 1(d)). The prognostic value of PTBP1 in SARC was further confirmed by Kaplan-Meier analysis, and the results showed a significant difference in OS and DSS between the low- and high-expression groups divided by median expression of PTBP1 (*P* < 0.05) (Figure 1(e)). The above results suggested that PTBP1 was upregulated in various tumors (e.g., SARC), and its high expression was correlated with poor prognosis.

### 3.2. Genetic Alteration of PTBP1

The cBioPortal website was used to explore the genetic alteration frequency of PTBP1 among different cancers (Figure 2(a), Supplement Figure 2A), and PTBP1 alterations most frequently occurred in SARC, followed by CESC, UCEC, OV, and LGG. The majority types of PTBP1 alterations in SARC included amplification, deep deletion, and mutation. Besides, a total of 104 mutation sites containing 77 missenses, 9 truncating, 15 splice, and 4 SV/fusion variants were located between amino acid 0 to 531 (Figure 2(b)).

Considering the prevalence of genetic alteration of PTPBP1 in SARC, SARC patients were assigned to high- and low-expression groups according to the level of the expression of PTBP1. The top 20 most frequently altered genes in each group were presented by waterfall plots (Figures 2(c) and 2(d)). TP53 alteration, with the missense variant as the major component, showed the highest frequency in both groups: 34% in the high-expression group and 41% in the low-expression group. TP53, ATRX (22%, 9%), TTN (14%, 10%), MUC16 (12%, 13%), and RB1 (8%, 10%) were found as top-five gene alterations in p53, mTOR, apoptosis, DNA replication, RNA polymerase, Wnt signaling, and Notch signaling pathway.

Accordingly, we hypothesize that PTBP1 mutational events occur in multiple tumors, particularly in SARC and may play critical roles in modulating cell cycle, tumorigenesis, and immunity.

### 3.3. Biological Function Analyses of PTBP1

KEGG and HALLMARK enrichment analysis was conducted to explore the biological function of PTBP1. We found that cell cycle-related pathways (e.g., cell cycle, DNA replication, ribosome, E2F targets, G2M checkpoint, and mitotic spindle), MYC targets, IL-17 signaling, and spliceosome pathway were most enriched in PTBP1 high-expression group (Figure 3(a), Supplement Figure 3A), while some metabolism-related pathways in PTBP1 low-expression group (Figure 3(b), Supplement Figure 3B). Thus, we deciphered that PTBP1 could mainly upregulate cell cycle at a pan-cancer level. Consistent trends were found when we focused on SARC separately. In SARC, PTBP1 activated signaling pathways (e.g., the E2F targets, MYC targets, G2M checkpoint, spliceosome, cell cycle, and TP53) by enrichment analysis of the HALLMARK (Figure 3(c)), KEGG (Figure 3(d)), and Reactome (Supplement Figure 3C) datasets.

We further explored the correlation between the expression of PTBP1 and well-recognized tumor-related pathways (e.g., TGFB, autophagy, and WNT). Since TGFB is an evolutionarily conserved signaling pathway regulating various cellular processes (e.g., proliferation, differentiation, apoptosis, inflammation, and fibrosis) [22], the correlation between the expression levels of PTBP1 and TGFB pathway-related genes in pan-cancer was analyzed (Figure 3(e)). Interestingly, nearly almost all TGFB-related genes showed significant positive correlations with PTBPT expression.

Autophagy plays an opposing environment-dependent role in cancer, and interventions to regulate autophagy have been proposed as an option for cancer treatment [23]. As depicted in Figure 3(f), the expression level of PTBP1 showed a significant positive correlation with nearly all autophagy-related genes in pan-cancer.

The similar results reemerged when we turned to WNT signaling pathway-related genes, which are known to control myriad biological phenomena throughout the development and adult life of all animals [24] (Supplement Figure 3D).

To sum up, PTBP1 upregulates cell cycle-related signaling pathways in SARC and pan-cancer and is closely and positively correlated with TGFB, autophagy, and WNT signaling pathways at the pan-cancer level.

### 3.4. Correlation between Tumor Immunity and the Expression of PTBP1 in Pan-Cancer

Tumor immune cell infiltration is an independent predictor of the tumor immune status and survival [25]. To further explore the correlation between PTBP1 and tumor immunity, immune checkpoint genes, neoantigens, tumor stromal, and immune cells in pan-cancer were analyzed.

Immune checkpoint plays an essential role in cancer immunotherapy (e.g., enhancing antitumor immune responses) using checkpoint inhibitors [26]. As depicted in Figure 4(a), the expression of PTBP1 was significantly correlated with the expression of most immune checkpoint genes including CD276 (B7-H3), NRP1, ADORA2A, TNFRSF4, TNFSF15, CD200, and CD80 in LGG, LIHC, KICH, KIRC, and KIRP. Notably, CD276 was found positively correlated with the expression of PTBP1 in pan-cancer. CD276 belongs to the immunoglobulin superfamily, and studies have shown that it may participate in the regulation of T-cell-mediated immune response and correlated with worse prognosis in cancer patients [27].

One of the promising advancements of immunotherapy is personalized vaccines designed to trigger de novo T cell responses against neoantigens [28]. The analyses of neoantigens may help find new targets for immunotherapy. We found that the expression level of PTBP1 showed a significant positive correlation with the number of neoantigens in LGG and UCEC, meanwhile, negatively and significantly in THCA (*P* < 0.05) (Figure 4(b)).

Roozendaal and Mebius [29] reported that in addition to providing structural support for lymphoid organs, stromal cells also influence immune cell differentiation and immune response. Hence, studying the composition of the tumor stromal can help further understand the tumor immune microenvironment. In this study, the expression of PTBP1 was simultaneously and positively correlated with ESTIMATEScore (Figure 4(c)), ImmuneScore (Supplement Figure 4A), and StromalScore (Supplement Figure 4B) in LGG, negatively in ACC, BLCA, BRCA, ESCA, GBM, LUAD, LUSC, PAAD, SARC, SKCM, STAD, TGCT, THCA, THYM, and UCEC. Taken together, the above results reveal that PTBP1 could upregulate immune response and positively correlated with stromal composition in LGG. It may function in a reverse way in various types of cancers, including SARC.

Subsequently, we utilized commonly recognized immune signatures to quantify the level of immune cell infiltration and analyzed its correlation with the expression of PTBP1 and found that the expression of PTBP1 has different correlations with immune cells in pan-cancer. It is consistent that PTBP1 is positively correlated with resting CD4 memory T cells, resting NK cells, and M0 macrophages, but negatively correlated with CD8 T cells, plasma, activated NK cells, and memory B cells (Figure 4(d)).

In addition, immunotherapy has significantly improved patient outcomes, but the occurrence of T-cell exhaustion seriously affects the therapeutic efficacy of immunotherapy [30]. Accordingly, we investigated the correlation between the expression level of PTBP1 and T-cell exhaustion-related markers (Supplement Figure 4C) and found that the expression of PTBP1 in SARC showed a significant positive correlation with the above T cell exhaustion markers, suggesting that the T-cell exhaustion phenomenon may be widely present in SARC patients with highly expressed PTBP1.

### 3.5. Immune Infiltration and PTBP1 in SARC

Despite the promising results of Chimeric Antigen Receptor (CAR) T Cell therapy in treating B-cell lymphoma and acute lymphoblastic leukemia [31], the clinical outcome in SARC patients remains unsatisfactory. The immune infiltration in SARC was further analyzed, and it was found that tumor development and progression were correlated with multiple genomic aberrations, which might affect tumor-infiltrating immune cells (TIICs).

In SARC, deep deletion of PTBP1 reduced infiltration of CD8+ T cell and neutrophil and arm-level deletion of PTBP1 significantly reduced the infiltration of CD4+ T cell and macrophage (Figure 5(a)). The analysis of the correlation between TIIC abundance and the expression of PTBP1 in SARC revealed that a high expression level of PTBP1 significantly increased the neutrophil abundance and decreased the abundance of dendritic cells (Figure 5(b)). In addition, a more detailed analysis of the correlation between the level of infiltration of different immune cell types and PTBP1 expression was performed (Figure 5(c)). We found that PTBP1 was positively correlated with type 2 T helper cell and memory B cell significantly, and contrary correlations were found in many immune cell types, such as activated B cell, mast cell, monocyte, and activated CD8 T cell (*P* < 0.05).

### 3.6. PTBP1 Affects TMB, MSI, MMR, and Methyltransferase Expression in Pan-Cancer

As a new pillar of modern cancer treatment, immunotherapy has revolutionized cancer management. TMB and MSI were taken as established immunotherapeutic response prediction in multiple tumor types [32]. TMB represents mutations in tumor cells (e.g., single nucleotide variations (SNVs) and small insertions/deletions (Indels)). MSI refers to a change in MS sequence length caused by an insertion or deletion mutation during DNA replication. We statistically analyzed the correlation of the expression of PTBP1 with TMB (Figure 6(a)) and MSI (Figure 6(b)) and found that PTBP1 was positively correlated with TMB and MSI both in LGG, LUAD, LUSC, SARC, STAD, and UCEC (*P* < 0.05).

MSI is a consequence of DNA MMR deficiency [33]. MMR gene mutations may cause DNA replication errors, higher somatic mutations, and tumorigenesis. Our correlation analysis revealed that the expression of PTBP1 was positively correlated with the level of MMR gene expression in pan-cancer (Figure 6(c)).

DNA methylation is a form of chemical modification of DNA capable of changing gene expression without altering the DNA sequence, which can be detected early, frequently, consistently, and in specific cell types in cancer [34]. Our circle visualization of correlation analysis revealed that DNA methylation transferases were positively correlated with the expression of PTBP1 in almost all tumors except UCS (Figure 6(d)).

An overview of the above findings demonstrated that PTBP1 could upregulate TMB, MSI, and MMR in various cancers and mediate DNA methylation in pan-cancer and SARC.

### 3.7. Expression Level of PTBP1 Affects Drug Sensitivity

Drug resistance remains a major factor limiting outcomes for cancer patients. Early chemo-therapeutics can achieve initial successes, whereas drug resistance may quickly develop, leading to disease relapse [35]. To find potential sensitive drug treatment targeting on PTBP1, we analyzed the correlation between the expression of PTBP1 and IC50 data collected from Cell Miner and GDSC databases. IC50 of cladribine, 5-fluoro deoxy uridine, clofarabine, gemcitabine, sapacitabine, methylprednisolone, nelarabine, fludarabine, and cytarabine showed significant positive correlations with the expression level of PTBP1 (Figure 7(a)). Besides, a comparison between PTBP1 high- and low-expression groups showed that IC50 of topotecan, panobinostat, irinotecan, PF2341066, paclitaxel, TKI258, TAE684, and L-685458 in PTBP1 high-expression group was significantly lower than that in PTBP1 low-expression group (Figure 7(b)). All the above results may provide new ideas for developing potential drugs relating to the expression of PTBP1 for treating cancers.

### 3.8. Clinical and In Vitro Validation of PTBP1 in Osteosarcoma

Osteosarcoma was the most common bone SARC, the most common primary bone malignancy in pediatric population. We divided osteosarcoma patients from TARGET database into PTBP1 high- and low-expression group (cutoff value = 6.740955, range 4.639331~8.184960). Kaplan-Meier analysis showed that PTBP1 correlated with poor prognosis of osteosarcoma (Figure 8(a)). Consistent with the RNA upregulation of PTBP1 in SARC from above analyses, IHC analyses were detected higher PTBP1 protein expression in human osteosarcoma lesions than in adjacent tissues (Figures 8(b) and 8(c)). Further, western blot assay revealed that PTBP1 was upregulated in human osteosarcoma cell lines compared with hBMSC (Figure 8(d)).

To further investigate the effect of the expression level of PTBP1 on tumor cell function in osteosarcoma, we constructed a PTBP1 knockout HOS (HOS-PTBP1-KO) cell line by CRISPR/Cas9 system. The mRNA expression (Figure 8(e)) and protein expression (Figure 8(f)) of PTBP1 were significantly downregulated in HOS-PTBP1-KO cell line compared with HOS wild-type (HOS-WT) cell line, which confirmed the knockout of PTBP1. Cell proliferation was significantly reduced in the HOS-PTBP1-KO group compared to the HOS-WT group since the 72 h. (Figure 8(g)). Transwell migration and invasion assay were performed to compare the cell migration and invasion ability. Knockout of PTBP1 could reduce the function of cell migration and invasion (Figure 8(h)).

Besides, given the significant correlation between the expression of PTBP1 and cell cycle pathway, FACS experiment was used to assess the cell cycle of HOS cell line with or without PTBP1 knockout (Supplement Figure 5). PTBP1 knockout induces osteosarcoma cells accumulate in G0/G1 phrases.

In brief, PTBP1 was overexpressed in osteosarcoma tumor tissues and cell lines and correlated with poor prognosis for osteosarcoma patients. Knockout of the expression of PTBP1 can reduce cell proliferation, migration, invasion, and significantly affect cell cycle in vitro.

## 4. Discussion

With the study of tumorigenesis and tumor immunity, immunotherapy has emerged as an encouraging and remarkable research field in oncology. Cancer immunotherapies are capable of adjusting the immune system to detect and attack cancer cells using immune checkpoint inhibitors and adoptive cell therapy. Research on the mechanism of tumor escape has changed the therapeutic prospect for various solid and hematologic malignancies [36]. Sarcoma, representing a heterogeneous group of cancers originating from the mesenchymal tissues, can be classified into soft-tissue sarcoma (STS) and bone sarcoma (BS). Most SARC are not sensitive to radiotherapy or chemotherapy and have a high recurrence or metastasis rate after local surgery [4]. Some preclinical trials on sarcoma immunotherapy showed a positive response of sarcoma to immunotherapy, thus allowing more researchers to focus on the immunotherapy of sarcoma [37]. However, there is still a long way to go before immunotherapy can be practically used for treating sarcoma.

PTBP1, a splicing factor involved in pre-mRNA processing, mRNA metabolism, and transport, plays a critical role in regulating alternative splicing events. Existing studies proved that PTBP1 plays an essential role in cancer progression by facilitating cell proliferation and migration of glioma [38], colorectal cancer [11], and breast cancer cells [39]. PTBP1 plays a role in various biological functions as a regulator in cancers (e.g., the regulation of tumorigenesis, glycolysis, apoptosis, invasion, and migration [40]). PTBP1 has gained prominence in cancer research due to its extensive biological functions, which is also expected to provide new insights into refractory tumor treatment, especially insensitive SARC treatment.

However, a systematic analysis of PTBP1 in pan-cancer should be urgently conducted, knowing that pan-cancer analysis can reveal similarities and differences in dysregulation of key biological processes in tumors [41], thus providing insights into cancer prevention and the design of novel therapeutic targets. This study aimed to explore the characteristic features and their potential roles of PTBP1 focused on SARC at a pan-cancer level.

It was found in this study that PTBP1 mRNA expression was increased in most tumor types. Survival analysis revealed that a high expression level of PTBP1 was mostly correlated with poor survival of OS, PFI, and DSS in pan-cancer. Specifically, a high expression level of PTBP1 was a risk factor in ACC, KICH, LGG, LIHC, LUAD, MESO, PRAD, SARC, SKCM, and UVM, and a protective factor in KIRC, OV, READ, and THYM. In conclusion, the above results suggest that TPBP1 is a potential prognostic biomarker in most cancer types. Existing studies proved that PTBP1 may prove to be a prognostic marker in multiple myeloma (MM), LUAD, BLCA, and KIRC [42–45], which is consistent with our conclusion.

Genetic alteration accumulation is considered to drive the progression of normal cells to invasive cancer and metastatic disease, through hyperplastic and dysplastic stages [46]. The genetic alteration of PTBP1, primarily composed of mutation, amplification, and multiple alteration, frequently occurs in SARC. As revealed by additional research of alterations in SARC, TP53, ATRX, TTN, MUC16, and RB1 were top-five altered genes in PTBP1-high and PTBP1-low groups of SARC with different frequencies and alteration types in composition, which were primarily correlated with p53, mTOR, apoptosis, DNA replication, RNA polymerase, Wnt, and Notch signaling pathway. Existing studies reported that TP53 plays an essential antitumor role in osteosarcoma, Ewing sarcoma, chondrosarcoma, rhabdomyosarcoma (RMS), leiomyosarcoma (LMS), synovial sarcoma, liposarcoma (LPS), angiosarcoma, and undifferentiated pleomorphic sarcoma (UPS) [47]. Novo therapeutics targeting TP53 require further attention and research.

In-depth mechanism research of PTBP1 revealed that PTBP1 was significantly correlated with the regulation of cell cycle, E2F targets, G2M checkpoint, MYC targets, DNA replication, ribosome, and spliceosome pathways in pan-cancer, suggesting that PTBP1 may play an important role in maintaining tumor cell viability to promote tumor proliferation. Similar results were found in SARC alone. Suckale et al. [48] demonstrated that PTBP1 was highly expressed in embryonic stem cells and throughout embryonic development, which suggested that PTBP1 plays an essential role in early embryonic development. Kang et al. [49] reported that PTBP1 was a positive regulator of human hepatocellular carcinoma growth by enhancing cyclin D3 translation, consequently facilitating cell cycle progression and tumor growth. PTBP1 was also found to increase RCC cell migration, invasion, proliferation, and angiogenesis via the hypoxia-inducible factor-1*α* pathway [45]. The above previous findings are consistent with our results. Thus, further research into new therapeutic approaches to tumor cell cycle regulation for SARC patients has great potential and significance.

We conducted correlation analyses between the expression level of PTBP1 and genes relating to the most popular pathways (e.g., TGFB, autophagy, and WNT pathway) and found that PTBP1 was positively correlated with almost all the genes of TGFB, autophagy, and WNT pathways in pan-cancer. Sheng et al. [50] reported that ST7 anti-sense RNA 1 overexpression could inhibit glioma progression by suppressing Wnt/*β*-catenin signaling by downregulating the expression of PTBP1. PTBP1 was also reported to regulate the phosphatase and tensin homolog-phosphatidylinositol-4,5-bisphosphate 3-kinase/protein kinase B (PTEN-PI3K/Akt) pathway and autophagy, thus inducing the proliferation, invasion, and metastasis of breast cancer cells [39]. However, there are rare studies on the mechanisms by which PTBP1 affects tumorigenesis and immunity. The results of this study may provide new insights into this field of research.

Despite the remarkable success of immunotherapy in several types of solid cancers (e.g., melanoma, nonsmall cell lung cancer, bladder cancer, and mismatch repair-deficient cancers) [51], the clinical outcomes of immunotherapy remain unsatisfactory in more types of cancers. One reason for this is the lack of discovery novo diagnosis and therapeutic targets due to poorly understood tumor-immune interactions in cancer. It is generally recognized that tumor immune cell infiltration is an independent predictor of the tumor immune status and survival, so a better understanding about the correlation between PTBP1 and tumor immune infiltration may provide new insights into the way PTBP1 affects tumor prognosis. Our studies have suggested that PTBP1 could upregulate or downregulate immune infiltration in various tumors, which might interpret why survival analysis showed different roles of PTBP1 in pan-cancer settings. The immune cell infiltration analysis of PTBP1 in SARC alone showed that high expression of PTBP1 could lower the abundance of immune infiltrates of most immune cell types significantly, except type 2 T helper cell and memory B cell, which may explain the poor prognosis in PTBP1 high-expression SARC patients.

MSI and TMB have been considered established biomarkers to assess the response to ICPIs in multiple tumor types [32]. We found that TMB and MSI showed a significant positive correlation with PTBP1 in LGG, LUAD, LUSC, SARC, STAD, and UCEC, and similar results were reported in MMR gene and DNA methyltransferase expression. Thus, abnormal expression of PTBP1 may contribute to tumorigenesis by increasing tumor mutation, impairing DNA damage repair function, and facilitating DNA methylation.

Drug resistance refers to an impairment to cancer therapy, and developing novel drugs against drug resistance is time-consuming and challenging. Drug repurposing is more economical based on existing research data. The process of repurposing can provide novel insights into disease pathogenesis and discover new opportunities for pharmaceutical interventions [52]. Since PTBP1 was found to be widely overexpressed in pan-cancer, correlated with worse outcomes, extensively involved in several well-known tumor pathways and regulation of tumor cell cycle, we suggested that PTBP1 might be a novo diagnosis and therapeutic target. Accordingly, we analyzed the correlation between PTBP1 and preclinical and clinical drugs to find potential therapeutic solutions for tumors. We identified a number of drugs with positive sensitivities consistent with the expression level of PTBP1, including topotecan, panobinostat, irinotecan, PF2341066, paclitaxel, TKI258, TAE684, and L-685458, which provides a selection of potential drugs for the pharmacotherapy of PTBP1 overexpressed tumors.

The further validation in osteosarcoma datasets of TARGET database suggested that PTBP1 is correlated with poor prognosis of osteosarcoma. Osteosarcoma tissue IHC staining and osteosarcoma cell line western blot analyses proved the overexpressed PTBP1 in tumor compared with normal tissues and cell line. PTBP1 knockout was also performed in HOS cell line by CRISPR/Cas9 system. CCK8, Transwell migration, invasion, and FACS experiments revealed that knockout PTBP1 could inhibit the cell proliferation, migration, and invasion and facilitate G0/G1 phrase accumulation of osteosarcoma.

However, there are some deficiencies of this study. TCGA-SARC dataset is mainly composed of soft tissue sarcoma, but there are differences between osteosarcoma and soft tissue sarcoma in pathophysiology and clinical features. In addition, the TARGET-OS dataset lacks multiomics data, so the dataset cannot be analyzed in depth.

## 5. Conclusion

This study revealed the prognostic value of PTBP1 in SARC and PTBP1 can promote cell proliferation, migration, invasion, and cell cycle in vitro experiments. Besides, PTBP1 was closely involved in cell cycle, TGFB, autophagy, and WNT pathways at a pan-cancer level. The high expression of PTBP1 is correlated with worse prognosis by mediating immune infiltration of cancer cells. The above findings may bring novel perspectives to the treatment of tumor patients.

## Figures and Tables

**Figure 1:** Expression level of PTBP1 in pan-caner. (a) Expression level of PTBP1 in 20 cancer types from Oncomine database. (b) Comparison of the expression of PTBP1 between tumor and normal tissues from TCGA database. (c) Comparison of the expression of PTBP1 between paired tumor and normal tissues of 22 cancer types from TCGA database. (d) The forest plots for OS, PFI, and DSS with HRs (log10) and 95% CI for 33 different cancer types. (e) Kaplan-Meier analysis of OS, DSS, and PFI in TCGA SARC patients stratified by different expression levels of PTBP1. ∗*P* < 0.05, ∗∗*P* < 0.01, ∗∗∗*P* < 0.001, and ∗∗∗∗*P* < 0.0001.

**Figure 2:** The genetic alterations of PTBP1 and correlations with mRNA expression. (a) Total genetic alterations of PTBP1 based on cBioPortal website. (b) Mutation diagram of PTBP1 in all cancer types across protein domains. (c) Waterfall of the top 20 mutated genes in PTBP1 high-expression group of the TCGA SARC cohort. (d) Waterfall of the top 20 mutated genes in PTBP1 low-expression group of the TCGA SARC cohort.

**Figure 3:** The biological function of PTBP1 in pan-cancer. (a, b) Gene set enrichment analysis of PTBP1-related signaling pathways in KEGG datasets at a pan-cancer level. (c) Bubble map of gene set enrichment analysis of PTBP1-related signaling pathways in HALLMARK datasets in TCGA SARC cohort. (d) Gene set enrichment analysis of PTBP1-related signaling pathways in KEGG datasets in TCGA SARC cohort. (e) Correlation between the expression of PTBP1 and TGFB pathway genes in pan-cancer. (f) Correlation between the expression of PTBP1 and autophagy pathway genes in pan-cancer.

**Figure 4:** Correlations between tumor immunity and the expression of PTBP1 in pan-cancer. (a) Correlations of the expression of PTBP1 with immune checkpoint genes. (b) Correlations of the expression of PTBP1 with neoantigens count. (c) Correlation between the expression of PTBP1 and ESTIMATEScore. (d) Correlations of the expression of PTBP1 with immune cell infiltration. ∗*P* < 0.05, ∗∗*P* < 0.01, and ∗∗∗*P* < 0.001.

**Figure 5:** Correlations between tumor immunity and the expression of PTBP1 in SARC. (a) Correlation of immune infiltrate level and different mutation subtypes among TCGA SARC cohort. (b) Correlation of the expression of PTBP1 and multiple immune cell infiltration in Timer database. (c) Correlations between the expression of PTBP1 and NES of 17 immune cells in TCGA SARC cohort. ∗*P* < 0.05, ∗∗*P* < 0.01, and ∗∗∗*P* < 0.001.

**Figure 6:** Correlations of PTBP1 with TMB, MSI, MMR, and DNA methyltransferases in pan-cancer. (a) Correlations of the expression of PTBP1 with TMB. (b) Correlations of the expression of PTBP1 with MSI. (c) Correlations of the expression of PTBP1 with five MMR-related genes. (d) Correlations of the expression of PTBP1 with four methyltransferases (DNMT1: red, DNMT2: blue, DNMT3A: green, and DNMT3B: purple). ∗*P* < 0.05, ∗∗*P* < 0.01, and ∗∗∗*P* < 0.001.

**Figure 7:** Correlation between PTBP1 and IC50 for different drugs. (a) Correlation analysis between the expression of PTBP1 and IC50 of cladribine, 5-fluorodeoxyuridine, clofarabine, gemcitabine, sapacitabine, methylprednisolone, nelarabine, fludarabine, and cytarabine in pan-cancer. *P* < 0.05 was considered as statistically significant. (b) Comparison of IC50 of topotecan, panobinostat, irinotecan, PF2341066, paclitaxel, TKI258, TAE684, L-685458, RAF265, sorafenib, PD-0332991, ZD-6474, nutlin-3, PLX4720, PHA-665752, AEW541, AZD0530, erlotinib, nilotinib, PD-0325901, AZD6244, LBW242, lapatinib, and 17-AAG between groups stratified by expression levels of PTBP1. ∗∗*P* < 0.01, ∗∗∗*P* < 0.001, and ∗∗∗∗*P* < 0.0001.

**Figure 8:** Clinical and vitro validation of PTBP1 in osteosarcoma. (a) Kaplan-Meier analysis of OS in TARGET osteosarcoma patients stratified by different expression levels of PTBP1. (b) Representative images of IHC staining of PTPB1 in human osteosarcoma tumors and adjacent tissues. Scale bar: 200/50 *μ*m. IHC score: 0, negative; 1, weakly positive; 2 moderately positive; 3 strongly positive staining. (c) Barplot of IHC score for PTBP1 protein level assessed by IHC assay. (d) Western blotting of PTBP1 protein expression in human osteosarcoma cell lines and hBMSC cell line. (e) RT-PCR result of PTBP1 gene expression in HOS-WT and HOS-PTBP1-KO cell line. (f) Western blotting of PTBP1 protein expression in HOS-WT and HOS-PTBP1-KO cell line. (g) Cell proliferation of HOS-WT and HOS-PTBP1-KO cell line. (h) Cell migration and invasion of HOS-WT and HOS-PTBP1-KO cell line. ∗∗∗*P* < 0.001, ∗∗∗∗*P* < 0.0001, scale bar: 100 *μ*m.

## Data Availability

The public data used to support the findings of this study are included within the article.

## Supplementary Materials

Supplementary Materials Supplementary 1. Supplement Figure 1: PTBP1 expression in patients with different AJCC clinical stages. Supplementary 2. Supplement Figure 2: the genetic alterations of PTBP1 and associations with mRNA expression. Supplementary 3. Supplement Figure 3: the biological function of PTBP1 in pan-cancer and SARC. Supplementary 4. Supplement Figure 4: correlations between tumor immunity and PTBP1 expression in pan-cancer. Supplementary 5. Supplement Figure 5: the flow cytometry analysis of cell cycle distribution.
